# The Application of Antimicrobial Photodynamic Therapy (aPDT) in the Treatment of Peri-Implantitis

**DOI:** 10.1155/2022/3547398

**Published:** 2022-05-12

**Authors:** Tianyuan Zhao, Jungyul Song, Yuzhuo Ping, Meihua Li

**Affiliations:** ^1^Department of Stomatology, The Second Hospital of Jilin University, Changchun 130041, China; ^2^The Affiliated Second Hospital of Jiamusi University, Jiamusi 154000, China

## Abstract

**Background:**

This literature review evaluates the mechanisms and efficacy of different types of antimicrobial photodynamic therapy (aPDT) for treating peri-implantitis by reviewing existing experimental studies to provide guidance for the clinical application of antibacterial photodynamic therapy (aPDT) in oral implants.

**Materials and Methods:**

From February 2001 to February 2021, we have collected 152 randomized controlled trials of aPDT for peri-implantitis by searching the experimental studies and clinical trials published in PubMed, Embase, Web of Science, and Google Scholar databases via online search. After screening the retrieved literature, we finally selected 10 statistically significant literature for evaluation and review.

**Results:**

Compared with the traditional nonsurgical treatment of peri-implantitis, the aPDT was superior to the traditional mechanical irrigation treatment group in terms of periodontal indexes PD, BOP, PLI, and postoperative effect, and the difference was statistically significant (*P* < 0.05). Furthermore, the combination of the aPDT and other treatments shows the synergistic antibacterial effect, signifying better clinical effect in many aspects (*P* < 0.05). In these 10 papers, by comparing the probe depth (PD), bleeding on probing (BOP), synosteosis, and periodontal pathogenic bacteria detection, etc., obtained after treating peri-implantitis by application of the antimicrobial photodynamic therapy, and using the SPSS data analysis software for statistical data processing, we found that the antimicrobial photodynamic therapy combined with other periodontal treatments has a more prominent postoperative effect. Meanwhile, the antibacterial photodynamic therapy with targeted action of photosensitizer has strong specificity to some bacteria, while the synthetic photosensitize for antibacterial photodynamic therapy can show good inactivation effect on broad-spectrum periodontal anaerobes without side effect.

**Conclusion:**

The experimental studies and clinical data of antibacterial photodynamic therapy for treating peri-implantitis show a good postoperative treatment effect. In addition, it did not develop resistance due to the use of antibiotic drugs. Owing to multiple advantages from combining antibacterial photodynamic therapy and other treatments, it is applicable for clinical treatment.

## 1. Introduction

Peri-implantitis is an inflammatory pathological state of the organism that occurs in the hard and soft tissues around the oral implants, whose clinical manifestations mainly involve the peripheral gingival soft tissues and alveolar bone, which may cause bleeding in the gingival soft tissues, broken and absorbed alveolar bone, and loosening implants and cause other risks. It is one of the main factors to cause the failure of implant operation [1].

According to current studies, some believes that it is the bacterial plaque that is the root cause of the peri-implantitis, while other studies have shown that patients with periodontal disease can also show the same pathogen groups around their own implants as those in periodontal disease, such as Staphylococcus aureus, Streptococcus, and subgingival with actinomycetes [2]. Therefore, the key point for treating peri-implantitis is that how we can accurately and effectively remove the pathogenic factors of bacteria plaque around the implant. At present, the commonly used clinical treatments include mechanical therapy, antibiotic drug therapy, laser therapy, and aPDT antimicrobial photodynamic therapy. According to the study by Persson et al., it shows that the metal scaler for scaling in mechanical treatment and ultrasound treatment may damage the implant's surface. This will accelerate the formation and accumulation of pathogenic factors of plaque after surgery [3]. For the treatment of peri-implantitis with antibiotic drug therapy, clinically, we mostly choose nitroimidazole, tetracycline, and other options for treatment. Minocycline hydrochloride is a broad-spectrum antibiotic and antibacterial spectrum that positively affects treating pathogens of peri-implantitis. A previous study shows that minocycline hydrochloride, as a sustained release for periodontal treatment, may positively affect periodontal tissue fiber regeneration. However, the therapeutic effect of long-term application of minocycline hydrochloride remains to be verified by experiments [4]. Currently, laser therapy is now being used as a safe and minimally invasive treatment for peri-implantitis, mainly including Nd:YAG laser, Er:YAG laser, and CO2 laser. According to some studies, the wavelength of Er:YAG laser is similar to that of the water and hydroxyl group, and the water molecules at the laser-irradiated place can fully absorb energy. The irradiated local area will not burn the tissue due to the high temperature; instead, the microblasting generated will effectively remove and cut the oral soft and hard tissue. The Er laser has a bacteriostatic and antiseptic effect on pathogenic bacteria caused by periodontal condition [5] and can effectively promote the regeneration of bone tissue. Meanwhile, according to the clinical trial report by Gaspirc and Skaleric, laser therapy versus conventional surgery for peri-implantitis, the former has shown a significant healing effect of periodontal soft and hard tissue [6].

Based on findings in recent years, antibacterial photodynamic therapy (aPDT) effectively treats a local microbial infection. For the pathogens, including Staphylococcus aureus, Pseudomonas aeruginosa, Porphyromonas gingivalis, and multidrug-resistant bacteria [7], Rajendran's literature shows that photodynamic therapy (PDT) uses photosensitizers to release free oxygen or free radicals under light irradiation to kill bacteria in tissues. This therapy is capable of selectively killing bacteria without causing damage to surrounding tissues [8]. Besides, PDT has the advantage that it will not produce drug resistance, and it can also be used as an auxiliary means of surgical treatment, reaching a better and ideal effect [9].

As a result, we searched the published experimental studies and clinical trials on PubMed, Embase, Web of Science, and Google databases and collected 152 randomized controlled trials of antibacterial photodynamic therapy (aPDT) for treating peri-implantitis. After screening, we selected 10 papers of statistical significance to go through the test for significance.

Given the lack of clarity related to the effectiveness of nonsurgical treatments, this study is made to conduct a systematic review of controlled and randomized clinical trials related to the efficacy of peri-implantitis and its different adjuvant therapies.

## 2. Methods and Materials (See Figure 1)

### 2.1. Method

We searched the literatures published on PubMed, Embase, Web of Science, and Google Scholar databases between 2001 and February 2021 and included the retrieved clinical studies on antimicrobial photodynamic therapy for the treatment of peri-implantitis. There are no obvious conflicts between the retrieved articles.

#### 2.1.1. Inclusion Criteria

1. Study on the clinical treatment of oral peri-implantitis
2. Clinical treatment and application of antibacterial photodynamic therapy
3. Clinical studies that have passed ethical review and have reliable data

#### 2.1.2. Exclusion Criteria

1. Experimental studies on peri-implantitis in animals
2. Existence of significant flaws and errors in the design of the implants used in the study
3. Clinical study on peri-implantitis leading to implant loss

### 2.2. Search Strategy

The search strategy applied was as follows: (((Periimplantitis OR periimplantitis OR peri-implantitis) OR (peri-implantitis or clinical periimplantitis)) AND (bone-to-implant contact)).

Animal studies were excluded and language limits (English) were imposed. The obtained results were combined with manual searches of the bibliographies of all full-text articles and related reviews selected from the electronic search.

## 3. Results

Among the 152 relevant articles, 10 articles passed the data analysis of the consistency test (Kappa = 1) after excluding the duplicates and articles failing to meet the inclusion conditions. We found that there was no conflict relationship among these 10 articles. The antibacterial photodynamic therapy group had different results from those obtained by the mechanical therapy and normal saline irrigation group in all clinical trials. A total of 481 patients and 663 implants were included (Table 1).

The reason why we excluded other literature is that only part of the antimicrobial photodynamic therapy for peri-implantitis is based on animal experiments, lacking clinical data support. In addition, in some literatures, peri-implantitis may be caused by improper design of implant surgery.

In the analysis of antimicrobial photodynamic therapy and mechanical irrigation debridement for peri-implantitis (Table 1), generally, we observed that after aPDT treatment, the periodontal indexes of peri-implantitis showed a tendency to return to normal, and the recovery effect was slightly different among the groups. SPSS was used for statistical analysis (*P* < 0.05), which showed statistical significant.

According to the studies by Rakašević et al., the clinical adhesion level (CAL) of the PDT group recovered more quickly after 3 months of treatment, showing a significant advantage over the 0.1% chlorhexidine gel group; the bleeding was significantly improved after treatment [11]. In parallel, the research of Ohba et al. also showed that the PDT group was significantly higher than the irrigating group at baseline and after the treatment, and the PDT group had a significant therapeutic effect on short-term peri-implantitis [15].

The photodynamic therapy for the treatment of peri-implantitis also has obvious advantages on periodontal pathogenic bacteria [20, 21]. According to the research of Caccianiga et al., photodynamic therapy was better at reducing trauma and pain while improving bacteria and inflammation [22]. After 6 months of treatment of peri-implantitis with the photodynamic therapy, the periodontitis decreased, so does the detection depth and detection bleeding, and a large number of bacteria decreased. Besides, the Actinobacillus actinomycetemcomitan (Aa) and Porphyromonas gingivalis (PG) decreased by more than 70% compared with the baseline period before the treatment. It is also proved that photodynamic therapy is a good adjunct option to surgical treatment for peri-implantitis. Albaker et al. pointed out in their study that the OFD group also had a better peri-implant effect in the early stage [13].

Meanwhile, in the study of Romeo et al., the recovery effect of the aPDT group was better than that of the traditional mechanical defibrillation group in terms of the periodontal probing depth (PD) of the implant after the treatment. The aPDT group at the end of treatment was statistically significant [10].

## 4. Discussion

We can compare a large number of literature studies in terms of the effects of antibacterial photodynamic therapy, traditional mechanical therapy, and drug therapy. Through a systematic review of the literature, we have collected reliability analysis of the efficacy of antimicrobial photodynamic therapy to treat peri-implantitis.

Abduljabbar compared it with traditional mechanical therapy; the photodynamic therapy was proven to have a more effective effect on the regulation of periodontal microflora, which also significantly improved the recovery of peri-implantitis soft and hard tissue [19].

For the application of the photodynamic therapy for peri-implantitis, the effect of treatment recovery also depends on the selected photosensitizer. In most cases, we use toluidine blue as a photosensitizer for antibacterial photodynamic therapy. Alqahtani et al. have achieved an ideal therapeutic effect using the toluidine blue photosensitizer in photodynamic therapy [14]. In addition, natural photosensitizer and synthetic photosensitizer materials are also available. However, due to the lack of clinical trial data, clinical trials are still needed to prove the reliability of these photosensitizers [23].

Since antimicrobial photodynamic therapy has been widely used for that treatment of peri-implantitis, a group of literature data showed that the antibacterial photodynamic therapy combined with traditional mechanical therapy for peri-implantitis is superior to a single treatment scheme [24]. The experiment of Caccianiga et al. also provides a new clinical treatment option for future treatment of peri-implantitis [22].

## 5. Conclusion

After the statistical analysis of retrieved literatures, the combined application of antibacterial photodynamic therapy and traditional mechanical treatment for peri-implantitis can achieve an obvious therapeutic effect [18]. Besides, the selection of photosensitizer in antibacterial photodynamic therapy will also affect the periodontal recovery effect of treatment. Therefore, we need more randomized controlled clinical trials to collect various pieces of evidences to determine the best treatment option for peri-implantitis.

## Figures and Tables

**Figure 1:** Flow diagram of searching processes and results. Ten articles met inclusion criteria and thus selected for inclusion in the systematic review.

**Table 1:** Clinical peri-implant parameters of subjects in randomized clinical trials comparing antibacterial photodynamic therapy with mechanical irrigation debridement for peri-implantitis treatment.

Authors	Population	Test group	Control group	Measures or percentages	
				Test group	Control group
1. Romeo et al. [10]	Individuals: 40 Implants: 123 Control: 59 Test: 63	Ultrasonic debridement and air polishing with a micronized glycine powder Implant debridement at sites with PD ≥4 mm was done with carbon fiber-reinforced plastic curettes Laser-assisted antimicrobial photodynamic therapy based on the HELBO protocol at implant sites with PD ≥4 mm	Piezoelectric ablator in combination with a special nonmetal tip Implant debridement at sites with PD ≥4 mm was done with carbon fiber-reinforced plastic curettes	PD: 5 mm; 3 mm; 2 mm; and 2 mm PLI: 60%; 11%; 17%; and 17% BOP: 100%; 20%; 10%; and 0% Analyses at baseline and 6, 12, and 24 weeks	PD: 5 mm; 3 mm; 2 mm; and 3 mm PLI: 62%; 12%; 21%; and 25% BOP: 100%; 35%; 20%; and 10% Analyses at baseline and 6, 12, and 24 weeks
2. Rakašević et al. [11]	Individuals: 40 Implants: 52 Control: 25 Test: 27	Photodynamic therapy	0.1% chlorhexidine gel followed by saline irrigation	PD: 5.74 ± 1.55 and 3.26 ± 0.79 CAL: 5.32 ± 1.36 and 3.35 ± 1.67 BOP: 28% and 5% Analyses at baseline and 3 mon	PD: 4.48 ± 1.08 and 2.86 ± 0.755 CAL: 4.63 ± 1.28 and 3.16 ± 1.25 BOP: 24% and12% Analyses at baseline and 3 mon
3. Schär et al. [12]	Individuals: 40 Implants: 107 Control: 37 Test: 70	Photodynamic therapy (PDT)	Local drug delivery (LDD)	PD: 4.19 ± 0.55; 3.92 ± 0.61; and 3.83 ± 0.58 PLI: 0.13 ± 0.21; 0.01 ± 0.04; and 0.00 ± 0.00 BOP: 4.03 ± 1.66; 2.26 ± 1.28; and 1.51 ± 1.41 Analyses at baseline, 3 mon, and 6 mon	PD: 4.39 ± 0.77; 3.93 ± 0.59; and 3.90 ± 0.78 PLI: 0.21 ± 0.27; 0.01 ± 0.04; and 0.03 ± 0.15 BOP: 4.41 ± 1.47; 2.20 ± 1.28; and 2.10 ± 1.55 Analyses at baseline, 3 mon, and 6 mon
4. Albaker et al. [13]	Individuals: 24 Implants: 24 Control: 13 Test: 11	Antimicrobial photodynamic therapy (aPDT) and open flap debridement (OFD)	Open flap debridement (OFD)	PI: 44.7 ± 8.2, 21.2 ± 5.9, and 16.4 ± 5.1 BOP: 35.9 ± 10.6, 24.3 ± 6.1, and 17.4 ± 5.5 PD: 5.2 ± 1.2, 3.9 ± 1.2, and 3.7 ± 1.1 CBL: 4.1 ± 1.4, 3.7 ± 1.3, and 3.4 ± 1.4 Analyses at baseline and 6 and12 mon	PI: 48.3 ± 9.6, 19.5 ± 6.3, and 11.6 ± 4.7 BOP: 26.5 ± 8.4, 21.6 ± 5.0, and 14.8 ± 3.1 PD: 5.4 ± 1.0, 4.1 ± 1.1, and 3.9 ± 1.1 CBL: 4.5 ± 1.5, 4.0 ± 1.4, and 3.8 ± 1.4 Analyses at baseline and 6 and 12 mon
5. Alqahtani et al. [14]	Individuals: 98 Implants: 98 Control: 49 Test: 49	Mechanical debridement and photodynamic therapy	Mechanical debridement	Test 1: cigarette smokers PI: 54.6 ± 12.2%, 31.3 ± 5.5%, and 46.5 ± 7.3% BOP: 12.7 ± 2.6%, 8.1 ± 1.2%, and 12.6 ± 3.8% PD: 5.2 ± 0.4 mm, 2.5 ± 0.2 mm, and 4.6 ± 0.2 mm CBL: 5.2 ± 0.3 mm, 5 ± 0.1 mm, and 5 ± 0.2 mm Test 2: waterpipe smokers PI: 52.3 ± 10.4%, 30.5 ± 4.2%, and 44.2 ± 4.8% BOP: 14.1 ± 1.8%, 9.3 ± 0.8%, and 13.3 ± 6.1% PD: 4.8 ± 0.2 mm, 2.6 ± 0.3 mm, 4.2 ± 0.3 mm CBL: 4.6 ± 0.3 mm, 4.6 ± 0.2 mm, 4.6 ± 0.2 mm Test 3: never smokers PI: 39.6 ± 6.7%, 12.4 ± 2.8%, and 14.1 ± 3.1% BOP: 44.1 ± 6.3%, 6.1 ± 1.2%, and 8.2 ± 1.5% PD: 4.5 ± 0.2 mm, 2.2 ± 0.4 mm, and 2.4 ± 0.5 mm CBL: 4.3 ± 0.2 mm, 3.7 ± 0.3 mm, and 3.3 ± 0.4 mm Analyses at baseline and 3 and 6 mon	Control 1: cigarette smokers PI: 54.6 ± 12.2%, 42.5 ± 7.9%, and 43.7 ± 8.2% BOP: 12.7 ± 2.6%, 11.2 ± 1.7%, and 13.5 ± 5.6% PD: 5.2 ± 0.4 mm, 4.6 ± 0.7 mm, and 4.4 ± 0.3 mm CBL: 5.2 ± 0.3 mm, 5 ± 0.2 mm, and 5.1 ± 0.3 mm Control 2: waterpipe smokers PI: 52.3 ± 10.4%, 42.1 ± 6.4%, and 40.6 ± 9.3% BOP: 14.1 ± 1.8%, 12.5 ± 1.6%, and 12.7 ± 5.5% PD: 4.8 ± 0.2 mm, 4.1 ± 0.5 mm, and 4 ± 0.6 mm CBL: 4.6 ± 0.3 mm, 4.6 ± 0.2 mm, and 4.7 ± 0.8 mm Control 3: never smokers PI: 39.6 ± 6.7%, 26.5 ± 5.7%, and 23.4 ± 3.5% BOP: 44.1 ± 6.3%, 20.9 ± 4.3%, and 20.8 ± 4.1% PD: 4.5 ± 0.2 mm, 3.9 ± 0.4 mm, and 2.6 ± 0.4 mm CBL: 4.3 ± 0.2 mm, 4.3 ± 0.3 mm, and 4.1 ± 0.2 mm Analyses at baseline and 3 and 6 mon
6. Ohba et al. [15]	Individuals:21 Implants: 25 Control: 13 Test: 12	Antimicrobial photodynamic therapy	Irrigation	BOP: 83.3% and 83.3% PI: 1.00 ± 0.74 and 0.67 ± 0.78 Analyses at baseline and after treatment	BOP: 92.3% and 84.6% PI: 0.92 ± 0.95 and 0.69 ± 0.85 Analyses at baseline and after treatment
7. Karimi et al. [16]	Individuals:10 Implants: 30 Control: 15 Test: 15	Closed surface scaling and photodynamic therapy	Closed surface scaling	PD: 5.36 ± 1.13, 3.75 ± 0.9, and 3.13 ± 0.54 CAL: 7.36 ± 1.57, 5.57 ± 1.09, 4.79 ± 1.36 Analyses at baseline and 1.5 and 3 mon	PD: 5.08 ± 1.47, 5.09 ± 1.5, and 5.08 ± 1.5 CAL: 7.16 ± 1.4, 7.17 ± 1.4, and 7.18 ± 1.4 Analyses at baseline and 1.5 and 3 mon
8. Almohareb et al. [17]	Individuals: 40 Implants: 79 Control: 36 Test: 43	Photodynamic therapy and mechanical debridement	Mechanical debridement	PD: 5.2 ± 2.0, 4.4 ± 1.1, and 3.8 ± 0.9 BOP: 45.3 ± 14.8, 27.2 ± 13.3, and 18.6 ± 7.9 Analyses at baseline and 6 and 12 mon	PD: 5.4 ± 2.1, 4.7 ± 1.0, and 4.1 ± 1.0 BOP: 43.8 ± 13.9, 29.7 ± 13.2, and 25.7 ± 8.1 Analyses at baseline and 6 and 12 mon
9. Al Rifaiy et al. [18]	Individuals: 38 Implants: 65 Control: 27 Test: 38	Photodynamic therapy and mechanical debridement	Mechanical debridement	PI: 51.1 ± 10.4 and 13.2 ± 3.4 BOP: 14.6 ± 3.1 and 11.7 ± 0.5 PD: 4.3 ± 0.8 and 2.1 ± 0.3 Analyses at baseline and 12 weeks	PI: 46.8 ± 7.9 and 27.5 ± 8.8 BOP: 9.2 ± 1.0 and 7.9 ± 0.2 PD: 4.5 ± 0.9 and 2.2 ± 0.5 Analyses at baseline and 12 weeks
10. Abduljabbar [19]	Individuals: 60 Implants: 60 Control: 30 Test: 30	Photodynamic therapy and mechanical debridement	Mechanical debridement	PD: 26.2 ± 3.7, 5.1 ± 0.8, and 8.8 ± 0.3 BOP: 30.3 ± 4.2, 8.2 ± 4.6, and 10.8 ± 0.6 Analyses at baseline and 3 and 6 mon	PD: 29.5 ± 2.4, 15.5 ± 1.4, and 10.7 ± 0.7 BOP: 35.7 ± 9.1, 18.1 ± 2.4, and 15.5 ± 1.3 Analyses at baseline and 3 and 6 mon
